# Clinical Efficacy of Laparoscopic Billroth II Subtotal Gastrectomy Plus Lienal Polypeptide Injection for Gastric Cancer

**DOI:** 10.1155/2022/5162225

**Published:** 2022-06-22

**Authors:** Wei Yan, Siqi Yan, Wu He

**Affiliations:** Department of Oncology, Jingzhou First People's Hospital, Jingzhou 434000, China

## Abstract

**Objective:**

To evaluate the clinical efficacy of laparoscopic Billroth II subtotal gastrectomy plus lienal polypeptide injection for gastric cancer.

**Methods:**

Between May 2018 and January 2021, 110 patients with gastric cancer treated in Jingzhou First People's Hospital were recruited and assigned via the random number table method to either an observation group or a control group, with 55 patients in each group. All patients received laparoscopic Billroth II subtotal gastrectomy, and the observation group additionally received lienal polypeptide injection. Outcome measures include surgical indexes, clinical efficacy, and adverse events.

**Results:**

The patients in the observation group had significantly less intraoperative hemorrhage volume, smaller surgical wounds, shorter time lapse before passing gas and hospital stay, and longer operation time than those in the control group (*P* < 0.001). The observation group showed significantly higher efficacy than the control group (*P*=0.001). The observation group had a significantly lower incidence of toxic side effects and adverse events than the control group (*P* < 0.05). After treatment, the CD3^+^ and CD4^+^ levels were significantly elevated and the CD8^+^ level was decreased, with higher CD3^+^ and CD4^+^ levels and lower CD8^+^ levels in the observation group than in the control group (*P* < 0.05).

**Conclusion:**

In the treatment of patients with gastric cancer, laparoscopic Billroth II subtotal gastrectomy plus lienal polypeptide injection features promising efficacy, improves the immune function of patients, effectively reduces the occurrence of toxic side effects and adverse reactions, with less trauma and rapid recovery, which shows good potential for use in clinical application.

## 1. Introduction

Gastric cancer is a malignant tumor that originates from the epithelium of the gastric mucosa and occurs mostly in people over 50 years of age. Gastric cancer ranks fourth in prevalence and second in mortality of all tumors worldwide. The main causes of gastric cancer include chronic inflammation, atrophic gastritis, atrophic gastritis with intestinal epithelial hyperplasia, and heterotypic hyperplasia, and other adverse factors include *Helicobacter pylori* infection, unhealthy diet, and poor environment conditions [1]. The majority of gastric cancer patients have no specific symptoms in the early stage, such as fullness and indigestion, which are similar to the symptoms of chronic gastric diseases such as gastritis and gastric ulcer and are prone to be overlooked. The common reasons for most gastric cancer cases attending the clinic are epigastric pain and weight loss, by which time the disease has usually progressed to the advanced stage [2]. Most patients with early-stage gastric cancer could obtain radical cure after surgery, while progressive-stage cancers require comprehensive treatment based on the pathological type and clinical stages of gastric cancer, such as surgery-based treatment with perioperative chemotherapy, radiotherapy, and biotargeted therapy so as to prolong patient survival and improve their survival quality [3]. Distal gastrectomy is one of the standard procedures for distal gastric cancer [4]. Billroth II subtotal gastrectomy is a modified version of Billroth I operation [5, 6], in which the residual stomach and the upper jejunum are anastomosed after major gastric resection, and the duodenum is sewn up [7]. However, traditional open surgery is highly traumatic, with high surgical risks and slow postoperative recovery. With the development of laparoscopic technology, laparoscopic radical gastric cancer treatment has been widely used in clinical practice [8]. Chemotherapy is commonly used postoperatively to eliminate small lesions and tumor cells that are unresectable, but it is associated with toxic side effects and leads to poor prognosis. The prognosis of gastric cancer is related to the pathological stage, site, tissue type, biological behavior, and therapeutic measures of gastric cancer [9]. Lienal polypeptide injection is a sterile aqueous solution of peptides, free amino acids, nucleic acids, and total sugars with a molecular weight of fewer than 6,000 daltons made from healthy calf spleen extracts, mostly used in primary and secondary cellular immunodeficiency diseases [10]. Studies have demonstrated its effectiveness in boosting immunity and improving physical weakness in postoperative or critically ill patients. It has been shown that traditional Chinese medicine (TCM) shows good potential in the treatment and prevention of tumors [4], which, as an adjuvant treatment, can curb the growth of tumor cells and attenuate the toxic effects of chemotherapy [5]. This study was conducted to evaluate the clinical efficacy of laparoscopic Billroth II subtotal gastrectomy plus lienal polypeptide injection in the treatment of gastric cancer and to provide clinical references for treatment.

## 2. Materials and Methods

### 2.1. Participants

Between May 2018 and January 2021, 110 patients with gastric cancer treated in Jingzhou First People's Hospital were recruited and assigned via the random number table method to either an observation group or a control group, with 55 patients in each group. All patients received Billroth II subtotal gastrectomy, and the observation group additionally received lienal polypeptide injection. The research was approved by the Ethics Committee of the Jingzhou First People's Hospital, Approval No. 833301–6/7.

### 2.2. Inclusion and Exclusion Criteria

#### 2.2.1. Inclusion criteria

Patients who met the relevant diagnostic criteria in the Gastric Cancer Diagnostic and Treatment Standard, with an expected survival of >3 months, with preoperative pathologically confirmed gastric cancer, with preoperative cTNM (UICC/AJCC 2016 gastric cancer staging) stage II to III, with the tumor located in the lower and middle part of the stomach, which was estimated to meet the requirement of distal radical resection range, with nonemergency surgery, without preoperative chemoradiotherapy, with American Society of Anesthesiology (ASA) classification I–III, and who provided written informed consent were included.

#### 2.2.2. Exclusion criteria

Patients who received preoperative radiotherapy, with allergies to study-related drugs or a history of related allergy, and with other malignant tumors were excluded.

### 2.3. Treatment Methods

Patients in both groups underwent pathological examination after admission and received surgery after confirmation of the diagnosis. Before surgery, patients in both groups received routine examinations, such as electrocardiogram, chest X-ray, coagulation analysis, routine blood and urine testing, whole abdominal computed tomography (CT) scan, and contrast CT scanning.

All the patients received laparoscopic Billroth II subtotal gastrectomy. The surgery was performed after the family signed the consent form for surgery and anesthesia. After preoperative routine disinfection and draping, with the patient in the supine position, gastrointestinal decompression was performed, followed by insertion of a gastric tube to establish a CO_2_ pneumoperitoneum, with a pneumoperitoneum pressure of 12–14 mm·Hg. An incision of 10 cm in length was made at the superior border of the umbilicus as the main operating port, and the secondary operating port was made 2 cm below the rib margin in the left and right anterior axillary lines and 2 cm above the midclavicular line in the left and right sides. A 5 cm Trocar was placed in the main and secondary operating ports, respectively. The lymph nodes were dissected as per the Guidelines for Operative Laparoscopic Gastric Cancer Surgery [11], the vagus nerve was severed, and the corresponding vessels were clamped and separated using peptide clips. The duodenum was severed 3 cm below the pylorus and the gastric body was disconnected 5 cm from the upper edge of the tumor through the main operating port, followed by sewing up the duodenum and the collection of the specimen [12, 13]. Billroth II anastomosis was performed. After lifting the transverse colon, Billroth II anastomosis of the residual stomach and jejunum was performed with a linear cutter, intermittent reinforcement sutures were performed on the plasma muscle layer, and a drainage tube was placed in the right anterior axillary line incision after surgery [14].

The SOX regimen (oxaliplatin/tegafur, gimeracil, and oteracil potassium capsules) was used for postoperative chemotherapy. The patients received 130 mg/m^2^ of oxaliplatin (Approval No. H20113281, Lianyungang Jereh Pharmaceutical Co. Ltd.) diluted in 500 mL of 5% glucose solution through intravenous infusion for 3 h. Tegafur, gimeracil, and oteracil potassium capsules (Approval No. H2130816, Taiho Pharmaceutical Co. Ltd., Tokushima Plant) were administered twice daily in the morning and the evening. The duration of treatment was two courses, with one course of 4 weeks.

Patients in the observation group additionally received 10 mL of lienal polypeptide injection (Approval No. H22026497, Jilin Fengsheng Pharmaceutical Co. Ltd.) diluted in 500 mL of 5% glucose solution daily using an intravenous drip pump (2C1009K, Baxter). The drug was discontinued after 1 week of administration for 3 weeks. The duration of treatment was two courses, with one course of 4 weeks.

### 2.4. TCM Adjuvant Therapy

The patient received Fuzi Lizhong decoction as adjuvant therapy, and the ingredients include Bupleuri Radix 10 g, Cyperi Rhizoma 10 g, Aurantii Fructus 10 g, Atractylodis Macrocephalae Rhizoma 10 g, Paeoniae Radix Alba 10 g, Chuanxiong Rhizoma 10 g, Pinelliae Rhizoma 10 g, *Oroxylum indicum* 6 g, Gardeniae Fructus 6 g, Amomi Fructus 4.5 g, and licorice root 3 g. The above herbs were decocted in 500 ml of water and 250 ml of filtrate was collected for oral administration, one dose daily, with a half dose administered in the morning and a half in the evening, respectively. The duration of treatment was two courses, with one course of 4 weeks.

### 2.5. Outcome Measures

The duration of follow-up was 6 months.

1. Surgical indices: the operation time, intraoperative bleeding, wound length, time lapse before anal exhaustion, and hospital stay of the two groups were recorded and compared.
2. Treatment efficacy: with reference to the Criteria for Evaluation of Therapeutic Efficacy of Solid Tumors, Response Evaluation Criteria in Solid Tumors (RECIST) [15], the efficacy was divided into complete remission (CR), partial remission (PR), stable disease (SD), and progressive disease (PD). CR: the lesion disappeared; PR: the lesion reduced by >30% in volume compared with that before treatment; SD: there was no significant change in lesion; PD: the lesion increased by >20% in volume compared with that before treatment. Total efficacy =  (CR + PR)/total number of cases × 100%.
3. Toxic side effects: with reference to the National Cancer Institute Common Terminology Criteria for Adverse Events (NCI-CTCAE), the occurrence of toxic side effects, including myelosuppression, neurological impairment, nausea and vomiting, and neutropenia, was recorded in all patients and compared between groups.
4. Immune function: the changes in CD3^+^, CD4^+^, and CD8^+^ levels of all patients before and after treatment were recorded in detail and compared between groups. 2 ml of fasting morning peripheral venous blood was collected from all patients and centrifuged to obtain the serum for the determination of T-lymphocyte subsets, and the absolute values of CD3^+^, CD4^+^, and CD8^+^ were measured by cell biopsies.
5. Adverse reactions: the occurrence of adverse reactions, including diarrhea, constipation, heartburn, and reflux gastritis, was recorded for all patients after surgery and compared between groups.

### 2.6. Statistical Analysis

The SPSS22.0 software was used for data analyses. The measurement data are expressed as (mean ± SD) and analyzed using the independent sample *t*-test. The count data are expressed as rates (%) and analyzed using the chi-square test. Differences were considered statistically significant at *P* < 0.05.

## 3. Results

### 3.1. Clinical Patient Profile

The patient characteristics were comparable between the two groups (*P* > 0.05) (Table 1).

### 3.2. Surgical Indices

The patients in the observation group had significantly less intraoperative hemorrhage volume, smaller surgical wounds, shorter time lapse before passing gas and hospital stay, and longer operation time ((127.71 ± 17.77) ml, (8.08 ± 1.37) cm, (2.71 ± 0.35) d, (7.73 ± 1.23) d, (211.15 ± 21.56) min) than those in the control group ((348.18 ± 25.96) ml, (17.23 ± 2.05) cm, (3.92 ± 0.88) d, (11.17 ± 1.85) d, (211.15 ± 21.56) min) (*P* < 0.05). (Table 2).

### 3.3. Treatment Efficacy

There were 12 (21.82%) cases of CR, 25 (45.45%) cases of PR, 13 (23.64%) cases of SD, and 5 (9.09%) cases of PD in the control group. There were 21 (38.18%) cases of CR, 30 (54.55%) cases of PR, 3 (5.45%) cases of SD, and 1 (1.82%) case of PD in the observation group. The observation group showed significantly higher efficacy (92.73%) than the control group (67.27%) (*P*=0.001) (Table 3).

### 3.4. Toxic Side Effects

There were 15 (27.27%) cases of myelosuppression, 13 (23.64%) cases of neurological impairment, 9 (16.36%) cases of nausea and vomiting, and 7 (12.73%) cases of neutropenia in the control group, and there were 2 (3.64%) cases of myelosuppression, 3 (5.45%) cases of neurological impairment, 2 (3.64%) cases of nausea and vomiting, and 1 (1.82%) case of neutropenia in the observation group. The observation group had a significantly lower incidence of adverse events than the control group (*P* < 0.05) (Table 4).

### 3.5. Immune Function

Before treatment, the two groups showed similar immune function parameters (*P* > 0.05). After treatment, the CD3^+^ and CD4^+^ levels were significantly elevated and the CD^8+^ level was decreased, with higher CD3^+^ and CD4^+^ levels and lower CD8^+^ levels in the observation group ((60.54 ± 9.12)%, (46.95 ± 5.08)%, (28.98 ± 4.45)%) than in the control group ((55.15 ± 8.95)%, (33.78 ± 5.37)%, (32.01 ± 4.18)%) (*P* < 0.001) (Table 5).

### 3.6. Adverse Events

There were 1 (1.82%) case of diarrhea, 2 (3.64%) cases of constipation, 3 (5.45%) cases of heartburn, and 2 (3.64%) cases of reflux gastritis. There were 8 (14.55%) cases of diarrhea, 6 (10.91%) cases of constipation, 7 (12.73%) cases of heartburn, and 9 (16.36%) cases of reflux gastritis. The observation group had a lower incidence of adverse events (14.55%) than the control group (54.55%) (*P* < 0.001) (Table 6).

## 4. Discussion

Radical gastric resection is currently the most effective treatment for gastric cancer [15], and with the development of minimally invasive surgery, laparoscopic radical gastric resection has been widely used for gastric cancer, in which the quality of gastrointestinal tract reconstruction is a key factor in determining patients' postoperative quality of life [16]. Billroth II subtotal gastrectomy enables radical resection of gastric tumors without concerns about anastomotic tension. Postoperative chemotherapy is usually adopted to remove unresectable tumor lesions and cells but may impair patient immunity. Lienal polypeptide injection features good tolerance, favorable efficacy, and a high safety profile in clinical applications [17].

The results of the present study showed that the patients in the observation group had less intraoperative hemorrhage volume, smaller surgical wounds, shorter time lapse before passing gas and hospital stay, and longer operation time than those in the control group. In distal gastric cancer surgery [18], the deep lesion site and special anatomical structure result in high difficulties in surgical operation and increase the operation time, which is consistent with the results of previous studies. Compared with traditional open surgery, laparoscopic Billroth II subtotal gastrectomy is less invasive, thereby reducing intraoperative bleeding, avoiding large exposure of abdominal organs to air, and shortening the time lapse before passing gas [19]. Relevant studies suggest that the SOX chemotherapy regimen is effective in the treatment of advanced gastric cancer by killing tumor cells, blocking malignant tumor DNA synthesis, and inhibiting cell lines to prevent cancer progression and spread. However, chemotherapy may result in collateral damage to adjacent normal cells and disrupt the immune function of the body, giving rise to a cascade of toxic side effects. In this study, TCM was employed as an adjuvant therapy to suppress tumor cells, which stimulates immune cells to recognize and engulf cancer cells by regulating the secretion of cytokines [13], thereby preventing recurrence and metastasis after resection of the primary lesion [14].

In the present study, after treatment, the CD^3+^ and CD^4+^ levels were significantly elevated and the CD^8+^ level was decreased, with higher CD^3+^ and CD^4+^ levels and lower CD^8+^ levels in the observation group than in the control group, and the observation group had fewer toxic side effects than the control group, indicating that laparoscopic Billroth II subtotal gastrectomy plus lienal polypeptide injection activates the nonspecific immune function of the body to improve the immunity, and the Fuzi Lizhong decoction contributes to enhancing the immunity of the body and attenuating the toxicity from chemotherapy. The reason may be that lienal polypeptide injection enters the spleen with blood circulation through an intravenous drip and improves immune cell activity through bidirectional multitarget immunomodulation, which enhances cellular nonspecific immune response and prevents serious toxic side effects. Previous research [20] suggests that lienal polypeptide injection has been widely used in postoperative chemotherapy for various cancers such as liver cancer and breast cancer with certain effectiveness, and the results of the present study also demonstrated its ability to mitigate the irritation of chemotherapy drugs on patients' gastrointestinal tract and effectively improve body immunity. Moreover, the observation group showed a significantly higher treatment efficacy and a lower incidence of adverse events than the control group. The reason may be that compared with conventional open surgery, laparoscopic Billroth II subtotal gastrectomy plus lienal polypeptide injection has a small incision, less intraoperative bleeding, and faster postoperative recovery, thereby effectively reducing the incidence of complications and improving the prognosis, with a high safety profile, which is similar to previous research results.

## Figures and Tables

**Table 1:** Patient characteristics (±*s*).

Group	*n*	Gender		Age (year, *x* ± *s*)	Body mass index (kg/m^2^, *x* ± *s*)	Tumor size	TNM stage	
		Male	Female				II	III
Control	55	38	17	51.03 ± 5.87	21.03 ± 2.61	4.39 ± 1.52	29	26
Observation	55	40	15	50.88 ± 6.13	20.96 ± 2.83	4.41 ± 1.37	28	27
*t/X* ^2^		2.638		0.131	0.135	0.072	1.454	
*P* value		0.435		0.896	0.893	0.943	0.357	

**Table 2:** Surgical indices (±*s*).

Group	*n*	Operation time (min)	Intraoperative hemorrhage (ml)	Surgical wound (cm)	Time lapse before passing gas (d)	Hospital stay (d)
Control	55	145.15 ± 20.51	348.18 ± 25.96	17.23 ± 2.05	3.92 ± 0.88	11.17 ± 1.85
Observation	55	211.15 ± 21.56	127.71 ± 17.77	8.08 ± 1.37	2.71 ± 0.35	7.73 ± 1.23
*t*		16.449	51.973	27.521	9.475	11.484
*P* value		<0.001	<0.001	<0.001	<0.001	<0.001

**Table 3:** Treatment efficacy (*n* (%)).

Group	*n*	CR	PR	SD	PD	Total efficacy
Control	55	12 (21.82)	25 (45.45)	13 (23.64)	5 (9.09)	37 (67.27)
Observation	55	21 (38.18)	30 (54.55)	3 (5.45)	1 (1.82)	51 (92.73)
*X* ^2^	—	—	—	—	—	11.136
*P* value	—	—	—	—	—	0.001

CR, complete remission; PR, partial remission; SD, stable disease; PD, progressive disease.

**Table 4:** Toxic side effects (*n* (%)).

Group	*n*	Myelosuppression	Neurological impairment	Nausea and vomiting	Neutropenia
Control	55	15 (27.27)	13 (23.64)	9 (16.36)	7 (12.73)
Observation	55	2 (3.64)	3 (5.45)	2 (3.64)	1 (1.82)
*X* ^2^		11.785	7.314	4.949	4.734
*P* value		0.001	0.003	0.026	0.030

**Table 5:** CD3^+^, CD4^+^, and CD8^+^ levels (%, ±*s*).

Group	*n*	CD3^+^		CD4^+^		CD8^+^	
		Before treatment	After treatment	Before treatment	After treatment	Before treatment	After treatment
Control	55	50.99 ± 8.36	55.15 ± 8.95^*∗*^	30.02 ± 4.87	33.78 ± 5.37^*∗*^	33.98 ± 4.99	32.01 ± 4.18^*∗*^
Observation	55	51.15 ± 8.45	60.54 ± 9.12^*∗*^	29.98 ± 5.45	46.95 ± 5.08^*∗*^	33.54 ± 5.15	28.98 ± 4.45^*∗*^
*t*	—	2.348	3.128	0.041	13.213	0.455	3.681
*P* value	—	0.921	0.002	0.967	<0.001	0.650	<0.001

A significant difference, ^*∗*^*P* < 0.05 in the comparison between the pretreatment and post-treatment results in the same group.

**Table 6:** Adverse events (*n *(%)).

Group	*n*	Diarrhea	Constipation	Heartburn	Reflux gastritis	Total incidence
Control	55	8 (14.55)	6 (10.91)	7 (12.73)	9 (16.36)	30 (54.55)
Observation	55	1 (1.82)	2 (3.64)	3 (5.45)	2 (3.64)	8 (14.55)
*X* ^2^	—	—	—	—	—	19.459
*P* value	—	—	—	—	—	<0.001

## Data Availability

All the data generated or analyzed during this study are included in this published article.
